# Effect of tissue factor knockdown on the growth, invasion, chemoresistance and apoptosis of human gastric cancer cells

**DOI:** 10.3892/etm.2014.1591

**Published:** 2014-02-28

**Authors:** YONG-JIANG YU, XU-DONG HOU, YU-MIN LI

**Affiliations:** 1 Department of General Surgery, The 1st Hospital of Lanzhou University, Lanzhou, Gansu 730000, P.R. China; 2 Department of General Surgery, The 2nd Hospital of Lanzhou University, Lanzhou, Gansu 730020, P.R. China

**Keywords:** SGC7901 gastric cancer, tissue factor, RNA interference

## Abstract

This study aimed to explore the role of tissue factor (TF) and evaluate its antitumor effects in the biological processes of gastric cancer cells using the application of RNA interference technology to silence TF in the SGC7901 gastric cancer cell line. Specific small interfering RNA (siRNA) designed for targeting human TF was transfected into SGC7901 cells. The expression levels of TF in the cells were detected by reverse transcription-polymerase chain reaction. Cell proliferation and chemosensitivity were measured by Cell Counting Kit-8. The metastatic potential of the SGC7901 cells was determined by Transwell experiments and wound-healing assays. Cell apoptosis was assessed by Annexin V-fluorescein isothiocyanate/propidium iodide double-staining method. The expression levels of TF mRNA were significantly reduced by the TF-siRNA in the SGC7901 cells, resulting in the suppression of cell proliferation, chemoresistance and invasion, and subsequently the induction of cell apoptosis. TF knockdown with siRNA inhibits the growth, invasion and chemoresistance and enhances the apoptosis of SGC7901 cells, providing a potential approach for gene therapy against human gastric cancer.

## Introduction

Gastric cancer is one of the most common types of cancer in the world, and in 2011 ~70% of all cases of gastric cancer occurred in developing countries (1). Metastasis is the most common cause of mortality of patients with gastric cancer, and one of the most common causes of mortality in patients who have undergone radical resection of gastric cancer (2). Tissue factor (TF), a 47-kDa transmembrane glycoprotein, primarily initiates the coagulation cascade through binding to activated factor VII (FVIIa). Previous studies have reported that TF is highly expressed in several types of tumor, including cancers of the pancreas, prostate, breast, colon and lung (3,4), and TF is detectable on the surface of tumor cells and TF-bearing microparticles (MPs) in the blood circulation which are shed from the cell surface (5,6). Furthermore, the expression levels of TF are correlated with tumor growth, angiogenesis and metastasis. Previous studies have suggested that TF plays an important role in the pulmonary metastasis of melanoma (7,8). However, to the best of our knowledge, no study thus far has reported the antitumor effects and antitumor mechanism of the inhibition of TF expression by small interfering RNA (siRNA) in gastric cancer.

In the present study, RNA interference (RNAi) technology was applied to silence the expression of TF in the SGC7901 gastric cancer cell line.

## Materials and methods

### Design and synthesis of specific siRNA

The mRNA sequence of the TF gene was obtained through the GenBank sequence search, then siRNA design software was used to design four TF-targeted siRNA sequences and a negative control siRNA sequence (Table I). To avoid the formation of a termination signal, TTDAAGAGA was inserted into the loop-stem structure of the short hairpin RNA (shRNA) template and the T6 structure was used as the transcription termination sequence. At the 5′ end of the sense strand template, CACC or CACCG, and a *Bas*I restriction site were added, and at the 5′ end of the antisense strand template, GATC and a *Bam*HI restriction site were added.

### Construction and connection of pGPU6/GFP/Neo-TF expression vector

The DNA oligonucleotide was dissolved with Tris-EDTA buffer (pH 8.0), and the oligonucleotide solutions of the corresponding sense and antisense strands were added. The pGPU6/GFP/Neo vector (2 μg) was subjected to agarose gel electrophoresis and recycled with a Takara DNA Purification kit, version 2.0 (Takara Bio Inc., Otsu, Shiga, Japan). The concentration was then diluted to 50 ng/μl for connection with the pGPU6/GFP/Neo-shRNA vector (Shanghai GenePharma Co., Ltd., Shanghai, China), and the connected product was transformed into *Escherichia coli* DH5α.

### Extraction and identification of positive clones

A monoclonal bacterial colony was selected, inoculated in 5 ml LB resistant medium and incubated in a 37°C incubation shaker overnight (4.44 × g). The plasmid was extracted with a plasmid extraction kit [Sangon Biotech (Shanghai) Co., Ltd., Shanghai, China]. *Bgl*II was used for mono-enzyme digestion to identify whether the targeted DNA fragment had been correctly connected to the pGPU6/GFP/Neo vector. Two recombinant plasmids, with the targeted fragment confirmed by mono-enzyme digestion, were randomly selected and sent to Sangon Biotech (Shanghai) Co., Ltd. for detection of the sequences, and the concentration and purity detection was performed on 1 μl plasmid with an automatic spectrophotometer.

### Cell culture and transfection

The SGC7901 gastric cancer cell line (stored in our laboratory) was reanimated and placed in 10% fetal bovine serum medium for cultivation and passage in a 37°C and 5% CO_2_ incubator. The cells in the logarithmic growth phase were obtained, trypsinized, vaccinated and cultivated in G418 complete medium, with the final concentrations of G418 as 800, 700, 600, 500, 400, 300 and 0 μg/ml to determine the minimum lethal concentration of G418. The cells were seeded in a six-well plate and cultured to 90–95% confluence, then Opti-MEM (Gibco-BRL, Carlsbad, CA, USA) was used to wash the cells twice. The lipofection method was used to transfect the recombinant and empty plasmids into the cells. An inverted fluorescence microscope was used to observe the results of transfection. RPMI-1640 medium was then added to the complete medium with the screened G418 concentration following the cultivation passage, and after one week, the G418 complete medium was changed to maintain the concentration at 600 μg/ml. When the control cells were all dead and the colonies were observable with the naked eye, the colonies were selected for detection.

### Reverse transcription-polymerase chain reaction (RT-PCR)

Following extraction, the total RNA was then reverse-transcribed into cDNA for RT-PCR. The primer sequences of GAPDH were as follows: Upstream, 5′-GCACCGTCAAGGCTGAGAAC-3′; and downstream, 5′-TGGTGAAGACGCCAGTGGA-3′; with the amplified fragment as 138 bp. The primer sequences of the TF gene were: Upstream, 5′-CTCCCGAACAGTTAACCGGAAG-3′; and downstream, 5′-GCCAGGATGATGACAAGGATGA-3′; with the amplified fragment as 136 bp. The PCR reaction conditions were as follows: 50 cycles, each with denaturation at 95°C for 30 sec, 95°C for 5 sec, 60°C for 34 sec, and extension at 95°C for 15 sec. Agarose gel electrophoresis (1.5%) was performed and the integrated optical density was obtained with an image analysis system (Bio-Rad, Philadelphia, PA, USA) for the semi-quantitative analysis.

### CCK-8 (Cell Counting Kit-8) determination of cell proliferation

Following conventional digestion, the cells in the logarithmic growth phase were used to prepare a 1×10^5^ cells/ml single cell suspension with 10% fetal bovine serum medium. The experiment was divided into the blank control group, the negative control group and the pGPU6/GFP/Neo/TF group, with four repeated wells for each group, and the final volume of the culture medium of each well was 200 μl. CCK-8 solution (10 μl; Beyotime Institute of Biotechnology, Shanghai, China) was added to each well after 24, 48 and 72 h of transfection and the cultivation was terminated after 2 h at 37°C. The detection wavelength was selected as 450 nm in the ELISA to measure the absorbance of each well, the results were recorded and the growth curve was drawn according to the time-absorbance value of each group to compare the difference between the proliferative capacity of the three groups.

### Chemotherapeutic drug resistance testing

Following conventional digestion, the cells in the logarithmic growth phase were used to prepare a 1×10^5^ cells/ml single cell suspension with 10% fetal bovine serum medium, and each well of a 96-well plate was inoculated with 100 μl. The chemotherapy drug oxaliplatin (Jiangsu Hengrui Medicine Co., Ltd., Jiangsu, China) was diluted in autoclaved saline and configured into the different working concentrations of 6.25, 12.5, 25, 50 and 100 μg/ml. Four repeated wells were set up for each group, with a final volume of 200 μl for each well, then incubated for 48 h prior to the addition of the different concentrations of oxaliplatin to each well for a further 48-h incubation. CCK-8 (10 μl) was added to each well and incubated 2 h prior to the termination of incubation. A wavelength of 450 nm was selected for the ELISA assay, and the absorbance values of each well were measured. The results recorded were used to calculate the growth inhibition rates of oxaliplatin towards the cells of each group. Inhibition (%) = (1- medication group/control group) × 100%.

### Transwell experiments

Matrigel gum (2 mg/ml; 15 μl) was added to each well of the Transwell chamber, and the gum was spread on the surface of the bottom membrane of the Transwell chamber. The base membrane was hydrated for the preparation of the single cell suspension. RPMI-1640 cell medium, containing 10% fetal bovine serum, was added to a 24-well plate, with 600 μl in each well. The cell suspension was added into the Transwell chamber, with 100 μl in each well, and each well was repeated in three wells. The chamber was immersed in the complete medium of the 24-well plate and incubated at 37°C and 5% CO_2_ for 24 h. The chamber was removed, rinsed with phosphate-buffered saline (PBS), fixed with methanol for 10 min, and then washed with PBS. Crystal violet staining was performed on the chamber, and then it was rinsed and dried. The number of nuclei on the bottom surface of the polyester film of the Transwell chamber was detected under a microscope at high magnification to determine the degrees of cellular invasion. Four view fields of the high magnification were randomly selected to count the number of nuclei and then the average number was calculated. The experiment was repeated three times.

### Wound-healing assay

The cells of each group were seeded in a fibronectin-pre-custodite 24-well plate, with six wells for each group and 4×10^5^ cells/well. The cells were cultured overnight to form cell monolayers, then a pipette was used to draw a dash-shaped horizontal wound along the bottom of the plate. Serum-free Dulbecco’s modified Eagle’s medium was used for cultivation. The cell motilities were observed at 0 and 24 h, and the distance from the starting point to the farthest migrated nucleus was calculated, with the result expressed as the mobility degree: The percentage of migration width to the original width. The experiment was repeated five times.

### Detection of apoptosis levels

The cells were transferred into a Falcon tube and rinsed with the pre-cold 1X PBS buffer twice (111 × g for 5 min). Subsequently, a 5×10^5^ cells/ml cell suspension was prepared with 1X binding buffer and then 5 μl Annexin V-fluorescein isothiocyanate was added. After 15 min, 10 μl propidium iodide was added and the suspension was incubated in the dark at room temperature for 15 min. Binding buffer (1X; 400 μl) was added to the suspension and it was gently vortexed. Flow cytometry was used to detect the results 1 h later.

### Statistical analysis

SPSS software package, version 17.0 (SPSS, Inc., Chicago, IL, USA) was used for the statistical analysis. The measured data are expressed as the mean ± standard deviation. One-way analysis of variance and intergroup Student-Newman-Keuls test were performed for the statistical analysis. P<0.05 was considered to indicate a statistically significant difference.

## Results

### Identification of the recombinant plasmid pGPU6/GFP/Neo/TF

The enzyme digestion results showed that the recombinant plasmid contained the *Bam*HI digestion site instead of the *Pst*I digestion site, while the empty vector contained the two sites. Therefore when using the restrictive endonucleases *Bam*HI and *Pst*I for the digestion, the restructured plasmid was digested with *Bam*HI and appeared in the linear form, while when digested by *Pst*I, no change was identified. The empty vector was digested by the two enzymes (*Bam*HI and *PstI*) and appeared in the linear form, indicating that all digested plasmids were the positive recombinant vectors. Liquid (20 μl) of each plasmid was obtained and delivered to the Shanghai Invitrogen Biotechnology Co., Ltd. (Shanghai, China) for sequence identification. The sequencing results showed that the synthesized plasmid sequences were correct and successfully cloned into the selected vector, and no presence of abnormal bases was detected (Figs. 1 and 2).

### Plasmid transfection and screening

A UV spectrophotometer was used to detect the concentration and purity of the extracted plasmid DNA, and the results were satisfactory for the subsequent transfection step. The medium, with the final concentration of G418 as 800, 700, 600, 500, 400, 300 and 0 μg/ml, was used for the cultivation, and the screening concentration of SGC7901 was determined as 600 μg/ml and the maintaining concentration as 300 μg/ml. During the stable transfection stage, cell death was observed three days after the addition of the screening concentration, appearing as cell contraction, rounding, floating and gathering into groups. On the 8th day, the majority of cells were observed as dead, and a small number of transfected cells remained. When switched to the medium with the maintaining concentration, these transfected cells restored growth and gradually formed positive clones. The expanded resistant clones were transferred to a new culture flask on approximately the 3rd week, and were cultured until the cells grew to 70–80% confluence. Following sub-cultivation, the cells became stably-transfected cells containing the hairpin-siRNA expression plasmid.

### Effect of time towards the cellular transfection rate

An inverted fluorescence microscope was used to observe the expression of the green fluorescent protein following transfection. With 4 μg DNA, the transfection rates of the SGC7901 cells [transfection rate (%) = fluorescent cells under the same view field/all cells under the same view field] at 24, 48 and 72 h were 25, 40 and 30%, respectively, and the transfection rate at 48 h was significantly higher than that at 24 h, while the rate decreased at 72 h.

### RT-PCR

RT-PCR was used to detect the expression levels of the TF gene, and the results showed that, compared with those of the control and negative control groups, the transfected expression levels of pGPU6/GFP/Neo/TF in each group decreased (P<0.05 or P<0.01). The expression levels of the TF-2 gene were the lowest, and the inhibitory effect was the most marked (P<0.01). Therefore, in subsequent experiments this was considered the experimental group. No significant difference in the expression levels of the TF gene was observed between the blank control and negative control groups (P>0.05; Table II).

### Inhibitory effect of TF-siRNA towards cell proliferation

The CCK-8 method was performed to detect the absorbance value A (the value is positively correlated with the number of viable cells) of each well of the blank control group, the negative control group and the experimental group at 24, 48 and 72 h. It was demonstrated that the levels of cell proliferation of the experimental group were significantly lower than those of the control group (P<0.05), while no significant difference between the blank control and negative control groups was identified (Fig. 3A).

### TF-siRNA reduces the chemotherapeutic drug resistance

A CCK-8 assay was used to detect the absorbance value of each group following the addition of oxaliplatin, and the inhibition rate was calculated. The results showed that the inhibition rate of oxaliplatin towards the pGPU6/GFP/Neo/TF-transfected cells was significantly higher than those of the control groups (P<0.05; Fig. 3B).

### Inhibition of TF-siRNA towards the cell invasion ability

To confirm the effect of TF-siRNA towards the migration and invasion of the tumor cells, a wound-healing assay and cell invasion experiment were performed on the SGC7901 gastric cancer cell line. As shown in Fig. 4, the wound-healing assay indicated that, compared with those of the negative control and blank control groups, the migration levels of the TF-siRNA group were significantly reduced (P<0.05). The results of the Transwell experiment showed that the cells of the three groups all passed through the Matrigel gel membrane. Compared with that of the negative control and blank control groups, the number of cells of the TF-siRNA group which penetrated the Matrigel gel membrane was significantly fewer (P<0.05), resulting in the significantly reduced invasiveness. These results suggested that TF-siRNA reduces the metastatic potential of gastric cancer cells.

### TF-siRNA increases the apoptosis of gastric cancer cells

To assess the induction towards apoptosis following the TF gene knockdown of SGC7901 gastric cancer cells, the double-staining method was performed to detect apoptosis 48 h after the transfection. The results showed that the percentage of apoptotic cells of the TF-siRNA group was 18.35%, significantly higher than that of the negative control (3.58%) and blank control (2.35%) groups (P<0.05), indicating that specific TF-siRNA may induce the apoptosis of tumor cells.

## Discussion

In normal tissue cells, the expression levels of TF are low or almost negative, but high expression levels of TF are detectable in a variety of types of solid malignant tumor. Previous studies have found that TF shows abnormal expression levels in various types of tumor cell, including gastric, colon and pancreatic cancer cells (9,10), and that its expression levels are closely associated with biological behaviors of tumor cells, including growth, invasion and metastasis, which were confirmed by the present study. *In vitro* and *in vivo* functional studies (11–13) have shown that TF significantly promotes tumor angiogenesis and enhances the invasion and metastasis abilities of tumor cells. In a previous study, a recombinant vector with the pcDNA3.1/TFcDNA plasmid was transfected into SGC7901 human gastric cancer cells, and the endogenous increased expression levels of TF significantly increased the levels of invasion and metastasis of the cells, and thus confirmed that TF was closely associated with the processes of invasion and metastasis of cancer (14). To further study the effects of the TF gene in the biological behaviors of gastric cancer, based on the high expression levels of TF in tumor cells and that siRNA efficiently inhibits the expression of the purpose gene, siRNA, which specifically encoded the TF gene, was designed, constructed, and transfected into SGC7901 gastric cancer cells to observe the siRNA-inhibited TF mRNA expression levels and function in the present study. It was demonstrated that the specifically targeted TF-siRNA effectively silenced the expression of the TF gene in SGC7901 human gastric cancer cells. The aforementioned method was used to study the changes in the biological behaviors of gastric cancer cells following TF knockdown. The expression levels of TF were correlated with the proliferative growth of the tumor cells (15). Through the CKK-8 method, it was observed that the growth of the gastric cancer cells was inhibited following the transfection of TF-siRNA *in vitro*, the inhibition was strongest after 48-h transfection, with an inhibition rate of 37%, and the cell proliferation ability significantly decreased. Following the chemotherapy of oxaliplatin, the inhibition rate of the gastric cancer cells significantly increased, indicating that following silencing of the TF gene, the growth of the gastric cancer cells was more likely to be suppressed by chemotherapy. Migration and invasion of tumor cells are the important steps in the process of tumor metastasis (16). The wound-healing assay and cell invasiveness test in the present study confirmed that TF-siRNA significantly reduced the potential migration and invasion effects of SGC7901 gastric cancer cells. These results suggested that TF is involved in coagulation and angiogenesis and plays an important role in the growth, invasion and metastasis of gastric cancer cells.

The effects of TF on tumor growth, invasion and metastasis are the joint action of its coagulation and non-coagulation pathways. Tumor cells themselves produce TF and stimulate the body to produce interleukin-1 (IL-1) and vascular endothelial growth factor (VEGF) (15). These procoagulant substances produce a hypercoagulable state within patients with tumors when they are exposed to endothelial cells and platelets *in vivo* (17). It has been reported that (18) the hypercoagulable state of patients with malignant tumors may depend on the TF-positive MPs in the circulation, and the MPs of different organizations are involved in the pathogenesis of tumor thrombus. In tumor-associated vascular diseases, the expression levels of TF in the circulation increase. For example, in human colon cancer, the TF in the circulation and on the membrane surface is associated with the occurrence of tumor cells and blood vessels (13). Tesselaar *et al* (19) also demonstrated that MP-associated TF was involved in the development of tumor-associated thrombosis in various types of adenocarcinoma.

Compared with those of the coagulation pathway, the functions of the TFs in the non-coagulation pathway are more important towards tumor invasion and metastasis. TF may promote tumor invasion and metastasis through intracellular signal transduction, regulating tumor angiogenesis and degrading the extracellular matrix (ECM), among other functions. In a previous study (20) it was shown that TF-FVII activates the signaling pathways of p44/42 mitogen-activated protein kinase (MAPK) and phosphatidylinositol 3 by activating protease activated receptor 2 (PAR2). TF-FVII may hydrolyze prothrombin, therefore hydrolyzing and activating the PARs, and then increasing the levels of cytokines, including IL-1β and IL-8 (21),. These factors may act as the messengers that regulate inflammation, and also stimulate the invasion and metastasis of tumor cells. The combination of TF and FVII may activate tyrosine kinase in the TF cell area, causing a Ca^2+^ influx, and then increase the transcription levels of VEGF through the MAPK or PKC signaling pathways. Numerous types of tumor have the activities of plasminogen activators, which is mainly caused by the increased activities of tissue plasminogen activator (PA) (22). The combination of TF and FVII was found to upregulate the expression levels of the urokinase PA in SW979 human pancreatic cancer cells, and it was thought that TF may increase the invasion and metastasis of tumor cells through upregulation the expression levels of plasminogen activator receptors (23). The plasmin activated by PA has high levels of proteolytic activity, which may degrade the ECM and thus promote tumor invasion and metastasis (24). Tumor cells not only secrete metalloproteinases (MMPs) by themselves, but also promote vascular endothelial cells to produce MMPs through secreting VEGF. They work together to degrade the basement membrane and ECM, and to stimulate the formation of new blood vessels (25). These pathways all promote the growth, invasion and metastasis of tumor cells.

Apoptosis inhibition is an important mechanism of tumorigenesis. The double staining method was used in the present study to detect the levels of apoptotic cells in each group, and demonstrated that the reduced expression levels of TF induced the apoptosis of SGC7901 gastric cancer cells. A study has shown that TF-FVII activates PI3K/Akt signal transduction to inhibit the doxorubicin-induced apoptosis in glioblastoma cells (26). Jiang, Guo and Bromberg (27) demonstrated that the complex of TF-FVII-factor X inhibits the apoptosis of breast cancer cells via the p44/42 MAPK and PKB/Akt signaling pathways. Whether or not its mechanism of apoptosis induction and its long-term silencing would lead to changes in the levels of anti-apoptotic factors requires further studies.

## Figures and Tables

**Figure 1:** Enzyme digestion identification of the recombinant plasmid. M, DNA marker. (A) The far left 1–5 lanes are the results of the TF-1 *Pst*I digestion; the next 1–5 lanes are the results of the TF-2 *Pst*I digestion; the following 1–5 lanes are the results of the TF-1 *Bam*HI digestion; and the far right 1–5 lanes are the results of the TF-2 *Bam*HI digestion. (B) The far left 1–5 lanes are the results of the TF-3 *Pst*I digestion; the next 1–5 lanes are the results of the TF-4 *Pst*I digestion; the following 1–5 lanes are the results of the TF-3 *Bam*HI digestion; and the far right 1–5 lanes are the results of the TF-4 *Bam*HI digestion. TF, tissue factor.

**Figure 2:** Sequencing of the recombinant plasmid. (A) pGPU6/GFP/Neo-TF1; (B) pGPU6/GFP/Neo-TF2; (C) pGPU6/GFP/Neo-TF3; and (D) pGPU6/GFP/Neo-TF4. TF, tissue factor.

**Figure 3:** (A) Cell growth curves of the different groups of cells prior to and following the transfection. Knockdown of TF with TF-siRNA inhibited cell proliferation of the gastric cancer cells *in vitro*. SGC7901 cell growth was significantly attenuated compared with that of the control and mock groups (P<0.05). (B) Inhibition rates of oxaliplatin towards the different groups. The inhibition rate of oxaliplatin towards the TF-siRNA-transfected SGC7901 cells was significantly higher than that of the the control and mock groups (P<0.05). TF, tissue factor; siRNA, small interfering RNA.

**Figure 4:** (A) Comparison of the *in vitro* migration degrees of the different groups. The bars represents the mean number of different cells. Knockdown of TF with TF-siRNA inhibited migration of the SGC7901 cells. P<0.05, versus the control and mock groups. (B) Comparison of the *in vitro* invasiveness of the different groups. The bars represents the mean number of cells per field. The invasion assay showed that knockdown of TF with TF-siRNA attenuated the invasion ability of the SGC7901 cells. P<0.05, versus the control and mock groups. TF, tissue factor; siRNA, small interfering RNA.

**Table I:** Interference fragment sequences of the TF gene.

Target gene	Sense sequence	Antisense sequence
TF-1	5′-CACCGCGCTTCAGGCACTAC AAATATTCAAGAGATATTTGTA GTGCCTGAAGCGCTTTTTTG-3′	5′-GATCCAAAAAAGCGCTTCAG GCACTACAAATATCTCTTGAAT ATTTGTAGTGCCTGAAGCGC-3′
TF-2	5′-CACCGGGAGCCTCTGTATGA GAACTTTCAAGAGAAGTTCTC ATACAGAGGCTCCCTTTTTTG-3′	5′-GATCCAAAAAAGGGAGCCT CTGTATGAGAACTTCTCTTGAA AGTTCTCATACAGAGGCTCCC-3′
TF-3	5′-CACCGGAACCCAAACCCGT CAATCATTCAAGAGATGATTGA CGGGTTTGGGTTCCTTTTTTG-3′	5′-GATCCAAAAAAGGAACCCA AACCCGTCAATCATCTCTTGAA TGATTGACGGGTTTGGGTTCC-3′
TF-4	5′-CACCGAATGTGACCGTAGA AGATGATTCAAGAGATCATCTT CTACGGTCACATTCTTTTTTG-3′	5′-GATCCAAAAAAGAATGTGA CCGTAGAAGATGATCTCTTGAA TCATCTTCTACGGTCACATTC-3′
Negative	5′-CACCGTTCTCCGAACGTGT CACGTCAAGAGATTACGTGAC ACGTTCGGAGAA TTTTTT	5′-GATCCAAAAAATTCTCCGA ACGTGTCACGTAATCTCTTGAC G-3′ GTGACACGTTCGGAGAAC-3′

TF, tissue factor.

**Table II:** Expression levels of the TF gene in SGC7901 gastric cancer cells.

Grouping	GAPDH Ct	TF Ct	ΔCt	ΔΔCt	2^−ΔΔCt^
N	32.95±0.55	23.87±0.04	−9.08±0.39	0	1
NC	32.77±0.03	23.85±0.32	−8.92±0.23	0.15717	0.864346
TF-1	31.86±1.08	26.13±0.21	−5.73±0.78	3.343803	0.483297^a^
TF-2	33.37±0.17	26.17±0.47	−7.2±0.37	1.875092	0.095393^b^
TF-3	32.34±0.82	24.25±0.43	−8.08±0.66	0.996823	0.310134^a^
TF-4	32.59±0.64	26.90±0.07	−5.69±0.45	3.389969	0.27261^a^

_Δ_Ct = TF Ct-GAPDH Ct, _ΔΔ_Ct = (TF Ct-GAPDH Ct) other samples - (TF Ct-GAPDH Ct).

a P<0.05, compared with the blank control group and the negative control group;

b P<0.01, compared with the blank control group and the negative control group.

TF, tissue factor; N, blank control; NC, negative control.
